# Imaging Diagnosis of Primary Liver Cancer Using Magnetic Resonance Dilated Weighted Imaging and the Treatment Effect of Sorafenib

**DOI:** 10.1155/2022/8586943

**Published:** 2022-06-28

**Authors:** Bin Fan, Yunyi Zhang, Shuai Guo

**Affiliations:** ^1^General Surgery, The First Affiliated Hospital of Northwest University (Xi'an No. 1 Hospital), Xi'an, 710000 Shaanxi, China; ^2^Public Health and Management Department, Ningxia Medical University, Yinchuan, 750001 Ningxia, China; ^3^Oncology Department, Huyi District People's Hospital, Xi'an, 710000 Shaanxi, China

## Abstract

**Objective:**

This work explores the application value of dilated weighted imaging (DWI) in the diagnosis of primary liver cancer (PLC) and the effect of sorafenib in the treatment of PLC.

**Methods:**

88 patients with PLC who were treated in The First Affiliated Hospital of Northwest University from March 2019 to March 2021 were selected and randomly rolled into an experimental group and a control group, with 44 cases in each group. Patients in both groups were treated with transcatheter arterial chemoembolization (TACE), and the patients in the experimental group were treated with oral sorafenib on the basis of TACE. The indicators of complications, short-term efficacy (STE), and long-term efficacy (LTE) of the two groups were observed. All patients received DWI and magnetic resonance (MR) plain scan. The diagnostic accuracy and misdiagnosis rate of the two methods in diagnosing the PLC were compared.

**Results:**

The accuracy, specificity, and sensitivity of MR plain scan were 68%, 88%, and 89%, respectively, while those of DWI were 96%, 95%, and 94.2%, respectively. It indicated that the accuracy, specificity, and sensitivity of DWI in diagnosing lesions were better than those of MR plain scan, especially the diagnostic accuracy (*P* < 0.05). The objective response rate (ORR) and disease control rate (DCR) of the STE in the experimental group were 30% and 97%, respectively, and those in the control group were 6% and 54.5%, respectively. The experimental group's mean progression-free survival (mPFS) and mean overall survival (mOS) were 12 and 25 months, respectively, while the control group's were 8 and 19 months, respectively. It was concluded that the mPFS and mOS of patients receiving TACE combined with oral sorafenib were much higher than those receiving TACE only (*P* < 0.05).

**Conclusion:**

DWI and TACE combined with sorafenib had high application value in the diagnosis and treatment of PLC.

## 1. Introduction

Primary liver cancer (PLC) is one of the malignant tumors with the highest incidence in the world. Clinical statistics show that 4.7% of new cancer patients are liver cancer patients each year, and liver cancer patients account for 8.2% of the number of cancer deaths each year. According to statistics from the World Health Organization (WHO), liver cancer has become one of the six major cancers in the world and the fourth leading cause of cancer-related death in 2018 [1–3]. The WHO also said that in the next few years, the incidence and death of liver cancer will continue to increase and rise. The incidence of liver cancer is affected by factors such as geographical location, ethnicity, economy, and food culture. Therefore, PLC has different incidence rates in different countries. Epidemiological survey results show that the incidence of PLC in Asia is relatively high, and the reason may be closely related to the relatively large population base in Asia [4]. The common cause of PLC is chronic liver disease caused by hepatitis virus. However, factors such as alcoholic liver disease, obesity, type 2 diabetes, and nonalcoholic fatty liver disease are also closely related to the occurrence of liver cancer. The main causes of liver cancer vary in different regions. In China, the biggest risk factors are hepatitis B infection and aflatoxin poisoning. Hepatitis C infection is the leading cause of death in Japan and Egypt. Obesity is the main reason for the increase in the incidence of liver cancer in areas with low incidence of liver cancer [5–7]. Epidemiological survey statistics show that the incidence of liver cancer in my country accounts for more than 50% of the world's, and liver cancer-related mortality ranks third in the world. At present, liver resection or liver transplantation is still the main method to ensure the long-term survival of PLC patients. However, clinical studies have shown that the early onset of PLC is relatively insidious, with no obvious clinical symptoms or even asymptomatic. This has led to the fact that most patients have already developed their disease in the middle and late stages when they come to see a doctor and have already lost the opportunity for surgical treatment. Clinical studies have shown that only less than 1/5 of patients can obtain the opportunity for surgery [8–10]. Despite the further development of medical technology in recent years, the treatment methods of PLC have gradually diversified. However, there is still no reliable and practical way for increasing patient survival rates. Liver cancer is characterised by a high blood supply, recurrence, and angiogenesis, according to clinical trials. Even in patients who have undergone surgical treatment, nearly 40% of patients relapse one year after surgery. 10% to 20% of patients have recurrence even after liver transplantation. China is a large hepatitis B country with a large population and a serious aging population. Generally speaking, the form of PLC is very serious [11].

Because PLC is usually found in the middle and late stages, many patients cannot be treated with surgery. Therefore, nonsurgical treatment is often used in the clinical treatment of PLC. Transcatheter arterial chemoembolization (TACE) is the most common treatment for hepatocellular carcinoma besides surgery. This method is to inject chemotherapy drugs such as doxorubicin, epirubicin, and cisplatin into tumor blood vessels and then embolize them with materials such as gelatin sponge [12]. The method has the advantages of less trauma, clear effect, wide application range, and high repeatability. However, this method also has some disadvantages, such as poor deposition of lipiodol and inability to completely embolize blood vessels. Based on the above shortcomings and the influence of the rich blood supply and angiogenesis of the PLC tumor itself, a single TACE treatment often fails to achieve the desired therapeutic effect. Therefore, TACE is often combined with other therapeutic methods to treat the PLC in clinical practice. Clinical studies have shown that TACE combined with systemic therapy can significantly prolong the survival of patients with advanced disease [13]. Sorafenib and apatinib are common oral targeted drugs in clinical practice. Among them, sorafenib is the first drug used in the systemic treatment of patients with advanced PLC and has shown good efficacy. It has been approved for first-line treatment of PLC. As an oral multienzyme inhibitor, sorafenib can act on tumor tissue and tissue blood vessels. It can block the formation of tumor angiogenesis, thereby inhibiting the growth of tumor tissue. Theoretically, the combination of TACE therapy and sorafenib can improve the prognosis of patients with advanced PLC. However, there is still a lack of effective large-scale clinical studies on this method, so further research is needed [14].

Computed tomography (CT) scan and enhancement, which can properly depict the number, size, shape, and deposition status of lipiodol, are currently the most effective and widely used procedures for the diagnosis and evaluation of the curative effect of PLC. However, due to the interference of high-density lipiodol, the density of the active tumor tissue lock may be misdiagnosed and missed. Ultrasound can observe the blood supply of tumors, but due to the influence of lipiodol, it is prone to chaotic strong echo reflections and limited spatial resolution of ultrasound [15]. Conventional magnetic resonance imaging (MRI) can detect tumor tissue but cannot differentiate between necrotic and viable parts. In recent years, magnetic resonance (MR) technology has developed rapidly. Some new technologies have been applied and developed, and people are gradually entering the era of diagnosing the PLC and evaluating the curative effect at the molecular level of functional status. Diffusion-weighted imaging (DWI) is one of them. DWI has a high sensitivity to Brownian motion of water molecules, and it is currently the only noninvasive method that can evaluate and identify the diffusion motion of water molecules in live tissue [16]. DWI can distinguish necrotic and residual viable tumor cells. The apparent diffusion coefficient (ADC) map can prove the signal difference between the two through quantitative analysis. The application of DWI technology may be able to solve the problem that conventional CT and MRI scans cannot quantitatively analyze tumor necrosis [17].

PLC patients were enrolled in this study and assigned to one of two groups: experimental or control. Patients in the experimental group received TACE in combination with sorafenib, while those in the control group received simply TACE. At the same time, all patients were diagnosed and evaluated by DWI technology, and the results were analyzed. This work is aimed at offering a reference and basis for clinical treatment and diagnosis of PLC.

The paper's organization paragraph is as follows: The materials and methods are presented in Section 2.  Section 3 presents the experimental results of the proposed work.  Section 4 consists of the discussion section. Finally, in Section 5, the research work is concluded.

## 2. Materials and Methods

### 2.1. Research Objects

88 PLC patients treated in The First Affiliated Hospital of Northwest University from March 2019 to March 2021 were selected, and they were rolled randomly into an experimental group and a control group, with 44 cases in each group. Patients included had to meet the following conditions: patients who were pathologically or clinically diagnosed as PLC, which could not be treated by surgery; patients with Barcelona liver cancer clinical stage (BCLC) of stage C; patients with estimated survival time of greater than 3 months; patients with no abnormality in blood routine, renal function, electrocardiogram, and other examinations before receiving treatment; and patients with no contraindications related to TACE and oral targeted drugs. Patients satisfying the below items had to be excluded: patients with or ever suffering from other malignant tumors; patients with severe liver damage; patients with severe heart, lung, kidney, or other systemic diseases; patients who received chemotherapy, radiotherapy, or other antitumor treatments; pregnant and breastfeeding females; and patients with a personal or family history of mental illness. All experiments in this work obtained patient informed consent and met the requirements of medical ethics.

### 2.2. Treatment Methods

All patients were treated with TACE. The patients in the experimental group were treated with oral sorafenib on the basis of TACE treatment. The detailed treatment process was as follows:

*TACE treatment*: angiography was performed through the celiac or common hepatic arteries using the Seldinger cannulation procedure. It could implant the catheter tip in the blood supply vessel, inject lipiodol and chemotherapeutic medications, and then employ gelatin sponge particles to embolize blood vessels once the tumor location, size, blood supply source, and other information were clearly understood. In addition, postoperative symptomatic and supportive treatment was performed. The specific dosage and treatment cycle of chemotherapeutic drugs were determined by the attending physician on the basis of the patient's review indicators.

*Sorafenib treatment*: the sorafenib tosylate tablets (Nexavar, Bayer Schering Pharmaceuticals, Imported Drug Registration Certificate No. H20160201, specification 0.2 g × 60 tablets/box, 5700 yuan/box) were adopted. The patient was required to take sorafenib tosylate tablets orally within 1 week after receiving TACE treatment, taking 0.4 g each time, twice a day. If any grade 3-4 adverse reactions related to medication occurred, the drug can be adjusted according to the specific situation of the patient. The dose was adjusted to 0.4 g/time, once a day.

### 2.3. MRI Examination

The instruments included GE Signa Excite 1.5 T superconducting MR scanner and 8-channel phased array soft body coil, TOSHIBA-SDF digital subtraction angiography system, and Marconi CT-Twin flash CT scanner.

The patient should fast for 6 hours prior to the assessment. The patient should practise holding their breath before the scan. All of the patients had standard MRI scans first, followed by T1WI cross-sectional suppression sequences, diffusion-weighted imaging, and finally cross-sectional dynamic contrast-enhanced images. The layer thickness of each sequence was 8 mm, layer spacing was 2 mm, field of view (FOV) was 34~40 c, and all were replicated to keep consistency. The specific imaging sequence and scanning parameters were as follows: FSPGR sequence T1WI: the time of repetition (TR) was 150 ms, time of echo (TE) was 4.2 ms, width of band (WB) was 41.7 kHz, flip angle was 85°, and matrix was 288 × 192. FRFSE (RT) sequence T2WI: TR was 6000 ms, TE was 87.1 ms, WB was 62.5 kHz, FOV was 34~40 cm, and matrix was 320 × 192. SE-EPI sequence diffusion-weighted imaging: TR was 1200 ms, TE was 59.0 ms, FOV was 35~38 cm, matrix was 128 × 128, number of excitations (NEX) was 4, and 3 different diffusion sensitivity factor *b* values were selected: 1000, 500, and 300 s/mm^2^ scan once each. At the same time, the diffusion gradient took three *X*, *Y*, and *Z* orientations. FSPGR sequence dynamic enhanced scan: TR was 125 ms, TE was 2.9 ms, WB was 83.33 kHz, FOV was 30~38, flip angle was 80°, and matrix was 288 × 192. The contrast agent was Gd~DTPA, the dose was calculated according to 0.2 mL/kg body weight, and the injection rate was 3 mL/s. After bolus injection through the antecubital vein, three rounds of sampling were performed at 15~18 s, 50~65 s, and 90~120 s, respectively.

### 2.4. Image Analysis and Judgment Criteria

Two experienced radiologists, combined with CT images, MRI plain scans, DWI images, and DSA angiography images, comprehensively analyzed the T1WI, T2WI, dynamic enhancement performance, and tumor blood supply staining to the necrosis, residual, and recurrence of the tumor. The results were compared with those of DWI images. The judging criteria were as follows. Residual tumor: after 1 month of treatment, MRI showed enhancement of the lesion, and DSA showed tumor staining. Tumor coagulation necrosis: after 1-3 months of treatment, MRI showed no enhancement of the lesion and no tumor staining on DSA. Tumor recurrence: new lesions appeared after complete necrosis of the tumor, MRI showed enhancement, and DSA showed tumor staining.

### 2.5. Evaluation of Treatment Effect

The patients were followed up by telephone, and the main items of follow-up were adverse reactions, liver-enhanced CT, DWI, and DSA angiography. The primary endpoint was OS. The measurement method of the maximum diameter of the target lesion in the same patient should be the same, and then, the RECIST1.1 standard was used to evaluate the efficacy of the patient. The specific efficacy evaluation methods are shown in Table 1.

### 2.6. Statistical Methods

All data analysis was completed by SPSS19.0. The measurement data were expressed in the form of mean ± standard deviation, and the test method was an independent sample *t*-test. The count data was expressed as frequency, and the comparison between groups was done by the chi-squared test. *P* < 0.05 meant the difference was statistically significant.

## 3. Results

### 3.1. General Data of Patients

Table 2 shows the general information for the two patient groups. It revealed that the experimental group consisted of 15 male and 19 female patients, with an average age of 48 years which was 55.3 ± 11.4, and the number of TACE times was 5.52 ± 3.88. The control group included 18 male patients and 14 female patients, the average age of the patients was 55.2 ± 12.2, and the number of TACE was 4.33 ± 4.13. The two groups of patients had no discernible differences in general data, and they were comparable.

### 3.2. Imaging Image Display of Typical Cases

The imaging images of typical cases are shown in Figure 1. It illustrated that the CT images of the patients generally showed round-shaped low-density lesions with a small amount of lipiodol deposition inside. MRI T1WI and T2WI lesions showed low T1WI and high T2WI signals. On dynamic contrast-enhanced magnetic resonance imaging, the lesions showed a marked enhancement in the arterial phase, and the enhancement in the portal venous phase and the delayed phase rapidly decreased and showed isointensity. DWI showed marked hyperintensity.

### 3.3. Correct Results of DWI in the Diagnosis of Various Lesions

The results of the correct diagnosis of the lesions are shown in Figure 2. It demonstrated that 90 lesions were found in this work, including 78 residual lesions, 6 lipiodol deposition lesions, 4 liquefaction lesions, and 2 coagulation necrosis lesions. 71 lesions were diagnosed by MR plain scan, including 62 residual lesions, 4 lipiodol deposition lesions, 3 liquefaction lesions, and 2 coagulation necrosis lesions. 89 lesions were diagnosed with DWI, including 76 residual lesions, 5 lipiodol deposition lesions, 5 liquefied lesions, and 3 coagulation necrosis lesions. The diagnostic results of the two methods were compared with the real data, the difference between the MR plain scan and the real data was large (*P* < 0.05), and the DWI diagnostic results were closer to the real data.  Figure 2(b) shows that the MR plain scan's accuracy, specificity, and sensitivity for diagnosing lesions were 68%, 88%, and 89%, respectively, whereas the DWI's accuracy, specificity, and sensitivity for diagnosing lesions were 96%, 95%, and 94.2%, respectively. It suggested that the accuracy, specificity, and sensitivity of DWI in diagnosing lesions were better than those of MR plain scan, especially that the accuracy was much better than that of MR plain scan (*P* < 0.05).

### 3.4. The Misdiagnosis of Lesions in Two Methods

The misdiagnosis of lesions by the two methods is shown in Figure 3. It revealed that the number of MR misdiagnosed lesions before treatment, 10 days, 30 days, 50 days, and 70 days of treatment was 0, 5, 7, 8, and 2, respectively. The number of DWI misdiagnosed lesions was 0, 2, 1, and 1, respectively. The number of DWI misdiagnosed lesions in each time period was less than that of MR plain scan (*P* < 0.05). The number of MR misdiagnosed lesions with diameters of 0-10 mm, 10-20 mm, 20-30 mm, 30-40 mm, and more than 40 mm was 3, 8, 5, 2, and 1, respectively. The number of misdiagnosed lesions on DWI was 1, 2, 0, 0, and 1, respectively. It meant that the number of lesions misdiagnosed on DWI was less than that on MR plain scan for lesions with different diameters (*P* < 0.05).

### 3.5. Comparison of STE between Two Groups of Patients

The comparison results of STE in the two groups of patients are shown in Figures 4 and 5. The numbers of CR, PR, SD, and PD patients in the experimental group were 2, 8, 33, and 1, respectively, and the ORR and DCR were 30% and 97%, respectively [18]. The numbers of CR, PR, SD, and PD patients in the control group were 0, 2, 22, and 20, respectively, and the ORR and DCR were 6% and 54.5%, respectively.

### 3.6. Comparison of LTE between Two Groups of Patients

Figures 6 and 7 show the LTE comparison results of the two groups of patients. The 6-month, 1-year, and 2-year survival rates of the experimental group were 95%, 68%, and 48%, respectively, while those in the control group were 86%, 53%, and 39%, respectively. Comparison showed that the survival rate of the experimental group in each time period was higher obviously than that of the control group (*P* < 0.05). The mPFS and mOS of the experimental group were 12 months and 25 months, respectively, while those were 8 months and 19 months, respectively, in the controls. The mPFS and mOS of the experimental group were greatly higher (*P* < 0.05).

### 3.7. Comparison on AFP

The AFP comparison results of the two groups of patients before and after treatment are shown in Figure 8. The figure illustrated that the pretreatment AFP of the experimental group and the control group was 715 and 697, respectively, and the posttreatment AFPs were 201 and 251, respectively. The intragroup comparison showed that the two groups of AFP were removed from the shelves after treatment, and the decrease in the experimental group was greater. No great difference in AFP was found between the two groups before treatment. After treatment, the AFP of the experimental group was remarkably higher.

### 3.8. Comparison of Complications between the Two Groups of Patients

The comparison results of complications between the two groups are shown in Figure 9. The number of patients in the experimental group with complications such as hand-foot syndrome, fatigue, hypertension, diarrhea, proteinuria, bone marrow suppression, and elevated transaminase was 1, 3, 0, 1, 0, and 1, respectively. The incidence of the disease was 13.6%. The number of patients in the control group with complications such as hand-foot syndrome, fatigue, hypertension, diarrhea, proteinuria, bone marrow suppression, and elevated transaminase was 2, 2, 1, 0, 0, and 2, respectively. The incidence of the disease was 15.9%. The difference in the incidence of complications was not obvious between the two groups.

## 4. Discussion

PLC is one of the common cancers that threaten human life and health. Clinical statistics show that the annual new cases of PLC in the world are 841,000, ranking 6th in the global incidence of malignant tumors, and the annual death cases are 781,000, ranking 4th in malignant tumors. In China, the proportion of new cases every year is 46.6%, and the proportion of deaths is 54.6%. In general, PLC has the characteristics of high malignancy, rapid progression, and insidious onset. It has caused a huge threat to the life safety of our people and also caused a huge economic burden [19].

At present, the common treatment methods for PLC include surgical treatment, local treatment, and systemic treatment. Surgery is still the main method for the treatment of PLC at present, and it is also the preferred treatment method for patients with PLC. Generally, liver resection and liver transplantation are commonly used. However, PLC has the characteristics of multicenter, which leads to the recurrence of nearly 40% of patients one year after surgery and more than 50% to 70% of patients after 5 years of surgery [20]. Even after liver transplantation, 10% to 20% of patients relapse. In addition, PLC also has the characteristics of insidious onset. Many patients have developed to the middle and late stages of PLC when they are diagnosed with PLC and have missed the opportunity for surgery and cannot be treated with surgery. For these patients, interventional therapy represented by TACE has become the preferred treatment method [18]. These methods have the advantages of minimally invasive, clear curative effect, and strong practicability, so they have been widely used in clinical practice. Numerous clinical studies have shown that TACE can significantly prolong the survival of patients, and the cumulative 1-, 3-, and 5-year survival rates are 57%-100%, 31%-52%, and 26%-34%, respectively. However, TACE embolization of blood vessels is not complete, so TACE is often combined with other treatment methods to treat liver cancer. Systemic therapy is the most prominent and most concerned area in clinical trials in recent years [21]. The efficacy of multikinase receptor inhibitors and monoclonal antibodies on advanced liver cancer has been confirmed. Sorafenib is the first targeted drug approved for the treatment of advanced liver cancer. Randomized double-blind trials in Europe, America, and Asia Pacific have confirmed that sorafenib can significantly prolong the effective survival of advanced liver cancer [22]. Scholars in North America, Europe, and Australia compared sorafenib with placebo, and the results showed that patients using sorafenib had a median overall survival improvement of 10.7 months compared with placebo, compared with 7.9 months for placebo; sorafenib also successfully extended patients' median progression-free time from 2.8 months to 5.5 months. Similar experiments were conducted in China and South Korea, again demonstrating the effectiveness of sorafenib. Theoretically, combining TACE with sorafenib could improve the survival rate of PLC patients. However, large-scale clinical studies are needed to confirm its efficacy [23, 24]. In this work, patients with PLC who missed the opportunity for surgery were selected as the research objects, and the patients were randomly rolled into an experimental group and a control group. The patients in the experimental group were treated with TACE+sorafenib, and the patients in the control group were treated with TACE alone. No obvious difference was found in the incidence of complications between the two groups, but both STE and LTE in the experimental group were significantly better. AFP decreased significantly more in the experimental group. This shows that the TACE+sorafenib treatment regimen can improve the survival rate and quality of life in patients with PLC effectively and greatly.

The most commonly used examination methods for the diagnosis and efficacy evaluation of PLC are CT scan and MRI. It can better detect and evaluate the number, size, shape, and lipiodol deposition of lesions. However, it also has certain defects. For example, under the influence of high-density lipiodol, the dominant density of some active tumor tissues is masked [25, 26]. Ultrasound and DSA have the disadvantage of not being able to assess the degree of tumor necrosis, and DSA is an invasive test. PET/CT has limited sensitivity and specificity. Compared with the above recurrence, MRI has the advantages of good tissue resolution, no radiation, and MRI signal not affected by lipiodol. It has gradually received extensive attention and application in the diagnosis and efficacy evaluation of liver cancer [27–29]. DWI can detect the motion state of water molecules in biological tissues, and the motion state of water molecules is closely related to tissue structure, biochemical properties, intracellular and extracellular volume changes, and extracellular space morphological changes. It can be said that this sequence can not only observe the morphological changes but also quantitatively analyze the tissue to achieve dual imaging of morphology and function [30]. Therefore, the introduction of DWI technology into the diagnosis of PLC may be able to achieve accurate qualitative analysis of PLC. In this work, DWI technology was introduced into the diagnosis of liver cancer patients, and its diagnostic effect was compared with the results of MR plain scan. The results suggested that the DWI diagnosis results were closer to the real data, and the misdiagnosis rate was lower. This shows that DWI diagnosis shows better performance in the diagnosis of PLC.

## 5. Conclusions

Patients with PLC who missed out on surgery were used as research subjects in this study, and they were assigned to the experimental and control groups at random. The patients in the experimental group were treated with TACE+sorafenib, and the patients in the control group were treated with TACE alone. Simultaneously, DWI technology was brought into the diagnosis of PLC patients, and its diagnostic effect was compared to that of an MR plain scan. According to the findings, there was no significant difference in the incidence of problems between the two groups, but the experimental group's STE and LTE were much better. In addition, AFP decreased significantly more in the experimental group. This shows that the TACE+sorafenib treatment regimen can improve the survival rate and quality of life in patients with PLC effectively. The DWI diagnosis results were closer to the real data, and the misdiagnosis rate was lower. To sum up, DWI had a good diagnostic efficiency for PLC, and TACE combined with sorafenib had a good therapeutic effect on PLC. There were still some limitations and shortcomings in this work. For example, it only compared the therapeutic effect of TACE alone and TACE combined with sorafenib. There was no comparison of the therapeutic effects of other medicines, such as apatinib coupled with TACE. As a result, the treatment technique suggested may not be the best option. Furthermore, only the findings of DWI and MR plain scan were compared and studied in the research on PLC diagnosis methods, in order to introduce more inspection methods. Failure to introduce more inspection methods may lead to insufficient objective and comprehensive research results. Future study and work would improve the above problems and conduct further in-depth research.

## Figures and Tables

**Figure 1:** Imaging images of typical cases.

**Figure 2:** Display of correct diagnosis results of lesions. Note: ∗ and # suggested *P* < 0.05 compared with the standard value and the MR plain scan, respectively.

**Figure 3:** The misdiagnosis of lesions of two methods. Note: ∗ meant *P* < 0.05 in contrast to DWI.

**Figure 4:** The number of patients in each stage of the two groups of patients. Note: ∗ meant *P* < 0.05 compared with the control group.

**Figure 5:** Comparison of ORR and DCR of patients. Note: ∗ meant *P* < 0.05 compared with the control group.

**Figure 6:** Survival rates of patients in the two groups at different time periods. Note: ∗ meant *P* < 0.05 compared with the control group.

**Figure 7:** Comparison of mPFS and mOS of patients. Note: ∗ meant *P* < 0.05 compared with the control group.

**Figure 8:** Comparison of AFP of patients. Note: # and ∗ meant *P* < 0.05 in contrast to the control group and the value before treatment, respectively.

**Figure 9:** Complications of the two groups of patients: (a) number of people; (b) proportion.

**Table 1:** Evaluation criteria of RECIST1.1.

Efficacy classification	Symptom descriptions
Progressive disease (PD)	The largest diameter and the lowest increase of the target lesion was ≥20% or the new lesion was found
Stable disease (SD)	The largest diameter and decrease in diameter of the target lesion did not reach PR or the enlargement diameter did not reach PD
Partial response (PR)	The largest diameter and decrease in diameter of the target lesion reached ≥30% and maintained for more than 4 weeks
Complete response (CR)	All target lesions disappeared, no new lesions appeared, and the tumor markers were normal and maintained for more than 4 weeks

Note: PR+CR was ORR; total DCR was the value of SD+PR+CR.

**Table 2:** General data of patients.

Indicator		Experimental group (*n* = 44)	Control group (*n* = 44)	*χ* ^2^/*t*	*P*
Age (years)		55.3 ± 11.4	55.2 ± 12.2	0.712	0.623

Gender	Males	15	18	—	—
	Females	19	14	—	—

Hepatitis B carriers				0.08	0.99
	Yes	25	26		
	No	19	18		

HBV replication				3.32	0.28
	Yes	20	23		
	No	24	21		

Vascular invasion				0.66	0.82
	Yes	21	17		
	No	23	27		

Distant metastasis				0.33	0.73
	Yes	25	23		
	No	19	21		

TACE times	5.52 ± 3.88	4.33 ± 4.13		0.068	1.03

## Data Availability

The data used to support the findings of this study are available from the corresponding author upon request.
